# Apple Peel Polyphenols and Their Beneficial Actions on Oxidative Stress and Inflammation

**DOI:** 10.1371/journal.pone.0053725

**Published:** 2013-01-23

**Authors:** Marie Claude Denis, Alexandra Furtos, Stéphanie Dudonné, Alain Montoudis, Carole Garofalo, Yves Desjardins, Edgard Delvin, Emile Levy

**Affiliations:** 1 Research Centre, Sainte-Justine Hospital, Montreal, Quebec, Canada; 2 Department of Nutrition, Faculty of Medicine, Université de Montréal, Montreal, Quebec, Canada; 3 Department of Biochemistry, Faculty of Medicine, Université de Montréal, Montreal, Quebec, Canada; 4 Institute of Nutraceuticals and Functional foods, Université Laval, Quebec, Quebec, Canada; Cordelier Research Center, France

## Abstract

Since gastrointestinal mucosa is constantly exposed to reactive oxygen species from various sources, the presence of antioxidants may contribute to the body’s natural defenses against inflammatory diseases.

**Hypothesis:**

To define the polyphenols extracted from dried apple peels (DAPP) and determine their antioxidant and anti-inflammatory potential in the intestine. Caco-2/15 cells were used to study the role of DAPP preventive actions against oxidative stress (OxS) and inflammation induced by iron-ascorbate (Fe/Asc) and lipopolysaccharide (LPS), respectively.

**Results:**

The combination of HPLC with fluorescence detection, HPLC-ESI-MS TOF and UPLC-ESI-MS/MS QQQ allowed us to characterize the phenolic compounds present in the DAPP (phenolic acids, flavonol glycosides, flavan-3-ols, procyanidins). The addition of Fe/Asc to Caco-2/15 cells induced OxS as demonstrated by the rise in malondialdehyde, depletion of n-3 polyunsaturated fatty acids, and alterations in the activity of endogenous antioxidants (SOD, GPx, G-Red). However, preincubation with DAPP prevented Fe/Asc-mediated lipid peroxidation and counteracted LPS-mediated inflammation as evidenced by the down-regulation of cytokines (TNF-α and IL-6), and prostaglandin E2. The mechanisms of action triggered by DAPP induced also a down-regulation of cyclooxygenase-2 and nuclear factor-κB, respectively. These actions were accompanied by the induction of Nrf2 (orchestrating cellular antioxidant defenses and maintaining redox homeostasis), and PGC-1α (the “master controller” of mitochondrial biogenesis).

**Conclusion:**

Our findings provide evidence of the capacity of DAPP to reduce OxS and inflammation, two pivotal processes involved in inflammatory bowel diseases.

## Introduction

Gastrointestinal mucosa is constantly exposed to luminal oxidants from ingested nutrients, such as alcohol, cholesterol oxides, and key among these is the simultaneous consumption of iron salts and ascorbic acid, which can cause oxidative damage to biomolecules [1], [2]. Moreover, local microbes or infections, ischemia/reperfusion, gastric acid production and nonsteroidal anti-inflammatory drugs may promote the formation of reactive radicals [3]–[5]. Additionally, the intestinal mucosa is subject to prolonged oxidative stress (OxS) from reactive oxygen species (ROS) generated during aerobic metabolism [6], [7]. The influx of neutrophils and monocytes associated with inflammation can further generate ROS via respiratory burst enzymes as well as those involved in prostaglandin and leukotriene metabolism [8]. Even if the etiology of inflammatory bowel diseases (IBD) has yet to be fully elucidated, a close relationship has been noted between ROS and the mucosal inflammatory process [9]–[13]. Although the specific events by which oxidants contribute to inflammation are not entirely elucidated, potential mechanisms include the activation of cyclooxygenage-2 (COX-2) and the transcription factor nuclear factor-kappa B (NF-κB) by pro-oxidants, thereby resulting in the initiation of the expression of genes controlling several aspects of the inflammatory, immune and acute phase responses [14]–[18].

Current epidemiological and experimental studies support a beneficial role of dietary polyphenols in several gastrointestinal diseases, including IBD [19]–[21]. Polyphenols are the most abundant antioxidants in the diet, (i.e. fruit, vegetables, beverages, herbs and spices) [22]–[26]. However, their poor intestinal absorption is responsible for luminal concentrations of phenolic compounds up to several hundred µmols in the gastrointestinal tract [27]. Most of these polyphenols exhibit powerful antioxidant activity by acting as free radical scavengers, hydrogen donating compounds, singlet oxygen quenchers and metal ion chelators, while they are also able to induce cellular antioxidant defense modulating protein and gene expressions [22], [24], [25], [28]. In the present investigation, we hypothesize that apple peel-derived polyphenols act in the gut as powerful antioxidants and anti-inflammatory agents capable of exerting protective effects against harmful intraluminal components in the gut, which may maintain the body’s natural defenses against a variety of intestinal diseases, including IBD.

## Materials and Methods

### Chemical and Reagents

HPLC-grade acetonitrile, methanol, acetone and Optima grade water were from Fisher Scientific (New Jersey, USA). Formic acid was purchased from Fluka (Steinheim, Germany). MTT was from Sigma (MO, USA). Apple peel crude extract (AB powder) and a purified polyphenolic fraction (JC-047) derived from dried apple peel powder (DAPP) were supplied from Leahy Orchards Inc. and AppleBoost Products Inc.

### DAPP Extraction

The phenolic compounds of apples (80% McIntosh and 20% a blend of Northern Spy, Cortland, Empire, Ida Red, Jonagold and Spartan) were extracted by a method similar to that reported previously by Liu’s laboratory [22], [29], [30]. Briefly, 25 g apple peels were blended with 200 g chilled 80% acetone solution in a Waring blender for 5 min. The sample was then homogenized for 3 min using a Virtis 45 homogenizer. The slurry was filtered through Whatman No. 1 filter paper in a Buchner funnel under vacuum. The solids were scraped into 150 g of 80% acetone and homogenized again for 3 min before refiltering. The filtrate was recovered and evaporated using a rotary evaporator at 45°C. This residue represented the apple peel crude extract (AB powder) while the purified polyphenolic fraction (JC-047) was isolated by preparative HPLC.

### LC-MS Analysis of DAPP Crude Extract and Purified Fraction

A reversed phase LC-MS method has been developed to separate and identify the mass and chemical structure of phenolic compounds derived from crude extract and purified fraction. Separations were performed on HPLC with fluorescence detection and HPLC-ESI-MS TOF (Agilent Technologies, Santa Clara, CA). The chromatographic column was a Halo C18, 3.0×100 mm, 2.7 µm particle sizes (Advanced Materials Technology Inc., Wilmington, DE) maintained at 50°C and operated at 0.3 mL/min. A two-step linear acetonitrile gradient was used for elution. The acetonitrile concentration was increased from 2 to 40% over 20 min then from 40 to 90% over the next 15 min followed by an equilibration step with the initial mobile phase composition for a total run time of 40 minutes. The mass spectrometer was operated in negative electrospray mode with a dual spray configuration allowing for internal calibration and therefore for a very good mass accuracy. This allowed us to extract narrow mass range peaks for quantitation purposes and increase the selectivity of the method. Mass spectra were acquired from m/z 100 to 2000 with an acquisition cycle of 0.89 s and a resolution greater than 10 000. The electrospray voltage was set at 3.5 kV, the fragmentor at 200 V and the source temperature at 300°C. Major phenolic compounds identified by HPLC-ESI-MS TOF were quantified by ultra-performance liquid chromatography system (UPLC) coupled to a tandem quadrupole mass spectrometer (MS/MS QQQ) equipped with an ESI source (UPLC-ESI-MS/MS QQQ). The UPLC-ESI-MS/MS QQQ system consisting of a Waters-ACQUITY UPLC with an AQUITY TDQ mass spectrometer (Waters, MA, USA). An Agilent Plus C18 column (2.1×100 mm, 1.8 µm particle sizes) (CA, USA) was used, and column temperature was maintained at 30°C. The phenolic compounds were separated using a gradient mobile phase consisted of 0.1% formic acid in ultrapure water and acetonitrile (solvent A and B respectively) with the flow rate of 0.4 µL/min. The following gradient was used: 0–8 min, 3–35% B; 8–9 min, 35–60% B; 9–10 min, 60–85% B; 10–11 min, 85% B; 11–11.10 min, 85–3% B; 11.10–14 min, 3% B. Data were acquired by MassLynx V4.1 software and processed for quantification with QuanLynx V4.1 (Waters, MA, USA). The UPLC-ESI-MS/MS QQQ system was operated with an ESI interface in negative ionization mode. Cone and collision gas flow rates, obtained from a nitrogen generator N2 were 80 L/h and 900 L/h, respectively. The mass spectrometer parameters were defined with Waters IntelliStart software (automatic tuning and calibration of the AQUITY TQD), and manually optimized as follow: capillary voltage of 3 kV, source temperature at 130°C and desolvation temperature at 400°C. Cone voltage was 30 V, and collision energy was 18 eV for all phenolic compounds. Quantification was determined using multiple reactions monitoring mode for all transitions of phenolic acids, flavonols, flavan-3-ols, procyanidins and dihydrochalcones.

### Determination of Total Phenolic Content of DAPP Crude Extract and Purified Fraction

The total phenolic content of AB powder or JC-047 fraction was determined using the Folin-Ciocalteu method [31], with gallic acid as a main standard. Briefly, 100 µL Folin-Ciocalteu reagent (diluted 10-fold in ultrapure water) and 80 µL sodium carbonate solution (7.5% in ultrapure water) were added to 20 µL MeOH (50% solution of extracts) in a 96-well plate. A blank sample and five calibration solutions of gallic acid (12.5 to 200 µg/mL) were analyzed under the same conditions. After 1 h-incubation at room temperature, the absorbance was measured at 765 nm using a Fisher Scientific Multiskan GO microplate reader (MA, USA). All determinations were carried out in triplicate and results were expressed as percentage of extract weight ± SEM.

### Heterogeneity of Fractionated Oligomers and Polymers of DAPP on Normal-phase HPLC

The procyanidin composition of AB powder and purified JC-047 fraction was analyzed as previously described [32] by normal phase analytical HPLC using an Agilent 1260/1290 Infinity system. Samples (5 µL of 25 mg/mL solutions in acetone/ultrapure water/acetic acid, 70∶29.5∶0.5) were injected into the HPLC system, and the separation was performed at 35°C with a flow rate of 0.8 mL/min using a Develosil Diol column (250 mm × 4.6 mm, 5 µm particle size), protected with a Cyano SecurityGuard column (Phenomenex, CA, USA). The elution was performed using a solvent system comprising solvents A (acetonitrile/acetic acid, 98∶2) and B (methanol/water/acetic acid, 95∶3∶2) mixed using a linear gradient from 0% to 40% B in 35 min, 40% to 100% B in 40 min, 100% isocratic B in 45 min and 100% to 0% B in 50 min. The column was re-equilibrated for 5 min between samples. Fluorescence of the procyanidins was monitored at excitation and emission wavelengths of 230 and 321 nm with the fluorescence detector, set to low sensitivity with a gain of 7X for the entire run. Individual procyanidins with DP from DP1 to DP>10 were quantified using an external calibration curve of (-)-epicatechin, taking into account their relative response factors in fluorescence [33]. The results were expressed as percentage of extract weight ± SEM.

### Intestinal Caco-2/15 Cell Culture

The human epithelial colorectal adenocarcinoma Caco-2/15 cell line, a stable clone of the parent Caco-2 cells (American Type Culture Collection, Rockville, MD), was obtained from Dr. JF Beaulieu (Department of Cellular Biology, Faculty of Medicine, Université de Sherbrooke, Sherbrooke, Quebec, Canada). Intestinal Caco-2/15 cells were cultured as described previously [34]–[42]. Briefly, they were grown in MEM supplemented with 10% decomplemented fetal bovine serum, 1% Penicillin-Streptomycin and 1% non-essential amino acids (all reagents from GIBCO-BRL, Grand Island, NY) at 37°C, 95% humidity and 5% CO_2_ as described previously [34]–[42]. Caco-2/15 cells were maintained in T-75 cm^2^ flasks (Corning Glass Works, Corning, NY) and were split (1∶5) when they reached 90% confluence using 0.05% trypsin-0.5 mM EDTA (GIBCO-BRL). For individual experiments, cells were plated at a density of 1×10^6^ cells/well on six-well culture plates, and were cultured for 10 days postconfluence, a period at which they are highly differentiated and appropriate for experimental treatments [34]–[42]. The medium was refreshed every second day.

### Caco-2/15 Cell Integrity

After various treatments, cell integrity was estimated by viability, morphology and differentiation assays. Briefly, cell differentiation was assessed by determination of villin protein expression. Monolayer intactness and physical barrier function were tested by evaluating morphology, transepithelial electric resistance and occludin protein expression. Finally, cell viability was appraised with 3-(4,5-dimethyldiazol-2-yl)-2,5 diphenyl Tetrazolium Bromid (MTT).

### Induction of Oxidative Stress and Inflammation

Differentiated intestinal Caco-2/15 cells were used to study the effects of the aforementioned polyphenols in OxS (Fe, 200 µM/Asc, 2 mM) and inflammation (LPS, 200 µg/mL) [41]. Crude extract (AB powder, 250 µg/mL) and purified (JC-047, 250 µg/mL) fraction were added to the apical compartment of Caco-2/15 cells for 24 h before incubation with iron/ascorbate (Fe/Asc) and/or lipopolysaccharide (LPS) for 6 h at 37°C. In order to distinguish between acute and chronic inflammation, Caco-2/15 cells were also incubated with LPS for a 24-h period. To highlight the mechanisms behind the beneficial actions of DAPP against OxS and inflammation, some experiments were carried out with 50 µM caffeic acid phenethyl ester (CAPE; Sigma, MO, USA) and 0.4 µM indomethacin heptyl esters (Cayman Chemical, Ann Arbor, MI) to inhibit NF-κB and COX-2, respectively.

### Lipid Peroxidation

Estimation of lipid peroxidation was assessed by measuring the release of malondialdehyde (MDA) from Caco-2/15 cells exposed to Fe/Asc (200 µM/2 mM) by HPLC. Briefly, proteins were precipitated with 8% sodium tungstate (Na_2_WO_4_) (Aldrich, Milwaukee, WI). The protein-free supernatants were then reacted with an equivalent volume of 0.5% (wt/vol) thiobarbituric acid solution (TBA; Sigma, MO, USA) at 95°C for 60 min. After cooling to room temperature, the pink chromogene [MDA-(TBA)_2_] was extracted with 1-butanol and dried over a stream of nitrogen at 50°C for 3 hours. The dry extract was then resuspended in 100% MeOH before MDA determination by HPLC with a fluorescence detection (Jasco Corporation, Tokyo, Japan) set at 515 nm excitation and 550 nm emission.

### Fatty Acid Analysis

Following differentiation, Caco-2/15 cells were incubated for 6 h at 37°C in the absence or presence of Fe/Asc (200 µM/2 mM), LPS (200 µg/mL) or both following pre-incubation with 250 µg/mL AB powder or JC-047 fraction, cells were then homogenized in PBS containing 0.005% (w/v) 2,6-Di-tert-butyl-4-methylphenol (Sigma, St-Louis, MO). Samples were subjected to transesterification and injected into a gas chromatograph using a 90 m×0.32 mm WCOT-fused silica capillary column VF-23 ms coated with 0.25 µm film thickness (Varian, Canada) according to the method described previously [43].

### Endogenous Antioxidant Enzyme Activities

Differentiated Caco-2/15 cells were harvested in hypotonic lysis buffer (10 mM HEPES, 1.5 mM MgCl_2_, 10 mM KCl, 0.5 mM DTT, 0.2 mM PMSF). Total superoxide dismutase (SOD) activity was determined as described by McCord *et al*. [44]. Briefly, superoxide radicals (O_2_^-^) were generated by the addition of xanthine and xanthine oxidase, and the oxidation of the SOD assay cocktail was followed using a spectrophotometer at 550 nm for 5 min. The same reaction was then repeated with the addition of the sample, and the SOD assay cocktail was less oxidized because of the SOD activity in the sample. The total SOD activity was then calculated. For glutathione peroxidase (GPx) activity, aliquots of cell homogenates were added to a PBS buffer containing 10 mM GSH, 0.1 U G-Red and 2 mM NADPH with 1.5% H_2_O_2_ to initiate the reaction. Absorbance was monitored every 30 sec at 340 nm for 5 min [41]. For G-Red activity, cell homogenates were added to a PBS buffer containing 2 mM NADPH and 10 mM of GSSG to initiate the reaction. Absorbance was monitored every 30 sec at 340 nm for 5 min [41].

### Immunoblot Analysis

Following the incubation with the various stimuli, differentiated Caco-2/15 cells were sonificated and the Bradford assay (Bio-Rad, Mississauga, Ontario) was used to determine the protein concentration of each sample. Proteins were denatured in sample buffer containing SDS and ß-mercaptoethanol, separated on a 7.5% SDS-PAGE and electroblotted onto Hybond nitrocellulose membranes (Amersham, Baie D’Urfé, Quebec, Canada). Signals were detected with an enhanced chemiluminescence system for antigen-antibody complexes. No specific binding sites of the membranes were blocked using defatted milk proteins followed by the addition of one of the following primary antibodies: 1/1000 polyclonal anti-villin (94 kDa; BD Biosciences, Mississauga, Ontario); 1/1000 polyclonal anti-occludin (59 kDa; Abcam, Campbridge, MA); 1∶1000 polyclonal anti-COX-2 (70 kDa; Novus, Oakville, ON); 1∶10000 polyclonal anti-NF-κB (65 kDa; Santa Cruz Biotechnology, Santa Cruz, CA); 1∶5000 polyclonal anti-IκB (39 kDa; Cell Signaling, Beverly MA); 1/5000 polyclonal anti- tumor necrosis factor (TNF)-α (26 kDa; R&D, Canada); 1/5000 monoclonal anti- interleukin (IL)-6 (25 kDa; R&D, Canada), 1/1000 polyclonal anti-Nrf2 (68 kDa; Abcam, MA, USA) and 1/1000 polyclonal anti-PGC-1α (92 kDa; Abcam, MA, USA), and 1∶40000 monoclonal anti-β-actin (42 kDa; Sigma, MO, USA).

The relative amount of primary antibody was detected with specie-specific horseradish peroxidase-conjugated secondary antibody (Jackson Laboratory, Bar Harbor, Maine). The β-actin protein expression was determined to confirm equal loading. Molecular size markers (Fermentas, Glen Burie, Maryland) were simultaneously loaded on gels. Blots were developed and the protein mass was quantitated by densitometry using an HP Scanjet scanner equipped with a transparency adapter and the UN-SCAN-IT gel 6.1 software.

### Prostaglandin E2 Determination

Cellular prostaglandin E2 (PGE2) was measured by enzyme-linked immunosorbent assay (Arbor Assay, Michigan, USA). After a short incubation, the reaction was stopped and the intensity of the generated color was detected in a microtiter plate reader (EnVision Multilabel Plate Readers, PerkinElmer) capable of measuring 450 nm wavelengths.

### Nuclear Extraction for Immunoblot Analysis of NF-κB, Nrf2 and PGC-1α

Differentiated Caco-2/15 cells were washed twice with PBS and left on ice for 4 min in a lysis buffer containing 10 mM HEPES, 10 mM KCl, 1.5 mM MgCl_2_, 2 mM DTT, and 0.4% Nonidet and antiproteases. Cells were then scraped and centrifuged for 5 min at 1,500 *g* at 4°C. Pellets were then washed with the same buffer, but without the Nonidet, and centrifuged again under the same conditions. The resulting pellets were then resuspended in 50 µL of final hypertonic lysis buffer (20 mM HEPES, 400 mM NaCl, 1.5 mM MgCl2, 0.2 mM EDTA, 2 1,4-dithio-DL-treitol, and 20% glycerol and antiproteases) and left on ice for 1 h with vortexing. They were then centrifuged for 10 min at 10,000 *g* at 4°C, and the supernatants were collected for protein and Western blotting to analyze NF-κB, nuclear factor erythroid-2-related factor 2 (Nrf2) and peroxisome proliferator-activated receptor gamma coactivator-1 alpha (PGC-1α) protein expression.

### Statistical Analysis

All values are expressed as mean ± SEM. Data were analyzed by using a one-way analysis variance and the two-tailed Student’s *t* test using the Prism 5.01 (GraphPad Software) and the differences between the means were assessed post-hoc using Tukey’s test. Statistical significance was defined as *P*<0.05.

## Results

### Profile of Phenolic Compounds of Crude and Purified DAPP

A reversed phase LC-MS method has been developed in order to separate and identify masses and chemical structures of polyphenolic compounds contained in the crude extract (AB powder) and purified polyphenol fraction (JC-047) derived from DAPP. Flavonoids figured among the major polyphenol classes: they were identified on the basis of their common structure consisting of two aromatic rings bound together by three carbon atoms that form an oxygenated heterocycle. Representative extracted ion chromatograms of identified polyphenolic compounds (using accurate mass measurement) are shown in Figures 1A and 2A. In the crude extract, flavonols constituted the dominant subclass of flavonoids and were present as a mixture of aglycone and glycosylated quercetin and dihydrochalcone (Figure 1B). Negative electrospray mass spectra of the deprotonated species [M-H]^-^ were observed [Table 1 and Figure 1C and at m/z 463,090 for quercetin 3-O-glucoside (1A); quercetin 3-O-galactoside (1B); m/z 433,079 for quercetin 3-O-arabinoside (1C); m/z 447,079 for quercetin 3-O-xyloside (1D); m/z 447,095 for quercetin 3-O-rhamnoside (1E) and m/z 435,131 for phloridzin (1F)]. On the other hand, the purified fraction was mainly composed of catechin, epicatechin and their oligomers eluting between 15 to 18 min (Figure 2B). Extracted ion chromatograms at m/z 289.076 are shown (+)-catechin eluting at 15.4 min and (−)-epicatechin eluting at 16.9 min (Figure 2B, left). The trimeric oligomers as proanthocyanidin trimer C1–C4 (Figure 2B, right) share the same m/z of 865.199 (Figure 2C). Colorimetric methods, including the Folin-Ciocalteu, were used for quantifying total phenolics content. The purified fraction contains a higher proportion (26%, *P*<0.01) of total phenolic compounds (1900±160 mg of gallic acid equivalents/100 g of extract weight) compared to the crude extract (1410±120 mg of gallic acid equivalents/100 g of extract weight). Furthermore, the combination of high performance liquid chromatography system (HPLC), coupled to a time-of-flight mass spectrometer (TOF) equipped with an HPLC-ESI-MS TOF; and UPLC-ESI-MS/MS QQQ analysis revealed higher amounts (mg/100 g) of flavonols+procyanidins and phenolic acids in purified JC-047 fraction compared to controls (137±9 vs. 369±10 and 74±1 vs. 43.0±6, respectively). However, the crude extract (AB powder) contained more flavonols and dihydrochalcones than the purified JC-047 fraction (346±14 vs. 207±16 and 261±6 vs. 255±11, respectively).

**Figure 1:** Separation and identification of polyphenolic compounds in DAPP crude AB powder. Extracted ion chromatograms of some identified polyphenolic compounds in AB powder using accurate mass measurement; (A). Extracted ion chromatograms of quercetin glycosides and dihydrochalcone (B) and their related mass spectra (C): quercetin 3-O-glucoside, m/z 463.0905 (1A); quercetin 3-O-galactoside, m/z 463.09018 (1B); quercetin 3-O-arabinoside, m/z 433.07914 (1C); quercetin 3-O-xyloside, m/z 447.07977 (1D); quercetin 3-O- rhamnoside, m/z 447.09506 (1E); and phloridzin, m/z 435.13171 (1F) obtained with negative ion electrospray ionisation. These polyphenols are provided from a mixture of 250 µg of crude extract DAPP in 1 mL Optima grade water.

**Figure 2:** Separation and identification of polyphenolic compounds in DAPP purified JC-047 fraction. Extracted ion chromatograms of some identified polyphenolic compounds in JC-047 using accurate mass measurement (A). Extracted ion chromatograms of catechin, epicatechin and trimeric flavan-3-ol oligomers C1 to C4 (B) and their related mass spectra (C): (+)-catechin, m/z 289.07541 (1A) and (-)-epicatechin, m/z 289.07659 (1B) and that trimeric flavan-3-ol oligomers C1 to C4 (2A to 2D) obtained with negative ion electrospray ionisation. These polyphenols provided of a mixture of 250 µg of purified fraction DAPP in 1 mL Optima grade water.

**Table 1:** Identification of procyanidins in DAPP.

AB powder		Formula	Ion formula[M-H]^-^	Experimentalmass (m/z)	Theoreticalmass (m/z)	Diff. ppm(<5 ppm)
Flavonols	Quercetin 3-O-glucoside	C_21_H_20_O_12_	C_21_H_19_O_12_	463,09050	463,08820	4.96
	Quercetin 3-O-galactoside	C_21_H_20_O_12_	C_21_H_19_O_12_	463,09018	463,08820	4.27
	Quercetin 3-O-arabinoside	C_20_H_18_O_11_	C_20_H_17_O_11_	433,07914	433,07763	3.47
	Quercetin 3-O-xyloside	C_20_H_18_O_11_	C_20_H_17_O_11_	433,07977	433,07763	4.92
	Quercetin 3-O-rhamnoside	C_21_H_20_O_11_	C_21_H_19_O_11_	447,09506	447,09329	3.96
Dihydrochalcone	Phloridzin	C_21_H_24_O_10_	C_21_H_23_O_10_	435,13171	435,12967	4.68

Experimental mass measurement and empirical formula calculation for quercetin glycosides and dihydrochalcone. A good agreement between the theoretical and the experimental m/z values was obtained for all compounds examined (<5 ppm). Separations were performed on an 1100 LC system coupled to an ESI-MSD-TOF mass spectrometer (Agilent Technologies, Santa Clara, CA).

The distribution of oligomers in the AB powder and JC-047 fraction was from degrees of polymerization (DP1 to DP10) [Table 2 and Figure 3]. However, the determination of total procyanidins content was 3 times higher in the JC-047 compared to the AB powder extract (Table 2)**.** No procyanidin oligomers higher than decamers were detected in the polymeric procyanidin signal.

**Figure 3:** Identification of procyanidins in DAPP. Representative chromatograms of DAPP (25 mg/mL) from AB powder (A) or JC-047 (B) were obtained by normal phase analytical HPLC using an Agilent 1260/1290 Infinity system coupled to a fluorescence detector.

**Table 2:** Heterogeneity of fractionated procyanidin oligomers and polymers of DAPP on normal-Phase HPLC.

Procyanidin content	DAPP (mg/100 g extract weight)	
	Crude extract (AB powder)	Purified fraction (JC-047)
Monomers	25.0±0.4	42.0±1.0***
Dimers	38.0±3.0	97.0±2.0***
Trimers	19.0±2.0	53.0±2.0***
Tetramers	13.0±1.0	46.0±1.0***
Pentamers	10.0±0.3	34.0±2.0***
Hexamers	9.0±1.0	29.0±2.0***
Heptamers	4.0±0.3	13.0±1.0*
Octamers	2.0±0.1	6.0±1.0
Nonamers	2.0±0.5	7.0±1.0
Decamers	1.0±1.0	2.0±0.5
Polymers DP>10	13.0±5.0	40.0±4.0***
**Total**	**137.0±9.0**	369.0±10.0***

The procyanidin composition of DAPP from 25 mg/mL crude extract (AB powder) and purified fraction (JC-047) was analyzed by normal phase analytical HPLC using an Agilent 1260/1290 Infinity system coupled to a fluorescence detector. Individual procyanidins with degrees of polymerization (DP) from DP1 to DP>10 were quantified using external calibration curve of (−)-epicatechin, taking into account their relative response factors in fluorescence. The results were expressed as mg/100 g of extract weight ± SEM. *P<0.05, ***P<0.001 vs. AB powder.

### Cell Integrity following Various Treatments

The effects of Fe/Asc and LPS on Caco-2/15 cells integrity were examined by morphology assessment, protein content quantification and MTT assay after incubation periods of 6 and 24 h. The morphology and the protein content remained unchanged with the administration of Fe/Asc, LPS and their combination, as well as following treatment with the AB powder or JC-047 (data not shown). Similarly, Caco-2/15 cell viability was not affected by the addition of the various treatments (Figure 4). Interestingly, an enhancement of villin protein mass was observed when Caco-2/15 cells were cultured in the presence of AB powder. Finally, there was no impact on Caco-2/15 cell monolayer transepithelial resistance (an indicator of cell confluence and monolayer integrity) (Figure 4) and on occludin protein mass (a biomarker for tight junction and mucosal barrier functions) (Figure 4). Therefore, it could be concluded that our experimental conditions, including the use of DAPP, did not exert any cytotoxic effects on Caco-2/15 cells.

**Figure 4:** Effects of DAPP on cell integrity in Caco-2/15 cells. Integrity of the monolayer was determined by cell viability, morphology (data not shown), differentiation and tight junction assays using fully differentiated Caco-2/15 cells. Crude AB powder (250 µg/mL) and purified JC-047 fraction (250 µg/mL) were added to the apical compartment of Caco-2/15 cells for 24 h before incubation with Fe/Asc (200 µM/2 mM) and LPS (200 µg/mL) for 6 h at 37°C as described in Materials and Methods. MTT (A), villin protein mass (B), transepithelial resistance (C) and occludin protein expression (D) were assessed. Results represent the means ± SEM of n = 3 independent experiments. *P<0.05 vs. Ctrl; ^##^ *P*<0.01 vs. Fe/Asc.

### Effects of DAPP on Lipid Peroxidation

The extent of lipid peroxidation following the treatment of Caco-2/15 cells with Fe/Asc during 6 h was assessed by determining cellular levels of MDA. HPLC analyses indicated a four-fold increase in MDA (*P*<0,001) following the administration of the oxygen free radical-generating system Fe/Asc compared to controls (Figure 5A). The presence of the AB powder or JC-047 fraction counteracted Fe/Asc-mediated lipid peroxidation with a more favorable impact of the former.

**Figure 5:** Effects of DAPP on lipid peroxidation and regulatory endogenous antioxidant activities in Caco-2/15 cells. Crude AB powder (250 µg/mL) and purified JC-047 fraction (250 µg/mL) were added to the apical compartment of differentiated Caco-2/15 cells for 24 h before incubation with Fe/Asc (200 µM/2 mM) and LPS (200 µg/mL) for 6 h at 37°C as described in Materials and Methods. Estimation of lipid peroxidation was assessed by measuring the MDA by HPLC (A). The activity of SOD (B), GPx (C) and G-Red (D) was then measured. Results represent the means ± SEM of n = 3 independent experiments. **P<0.01, ***P<0.001 vs. Ctrl; ^#^ *P*<0.05, ^##^ *P*<0.01, ^###^ *P*<0.001 vs. Fe/Asc; ^$$^ *P*<0.01, ^$$$^ *P*<0.001 vs. Fe/Asc+LPS.

Since OxS markedly altered the composition and properties of the bilayer lipid environment, we determined the profile of fatty acids (FA). In fact, the addition of Fe/Asc resulted in substantial differences in FA following the 6 h-period of cell incubation (Table 3). In particular, a significant decrease was noted in n-3 and n-6 polyunsaturated fatty acids (PUFA) (EPA, 20∶5n-3; DHA, 22∶6n-3; AA 20∶4n-6) as well as in monounsaturated FAs (18∶1n-9) (Table 2). As a consequence, the calculated total n-3, n-6 and n-9 was reduced by 3-fold, 0.5-fold and 2-fold compared to controls (Table 3). As n-3 FAs were more affected by OxS than n-6 FAs, a decline was recorded in the ratio n-6/n-3, which indicates an inflammatory state. Nevertheless, preincubation with the AB powder or JC-047 fraction restored the levels and composition of PUFAs.

**Table 3:** Effects of DAPP on fatty acid composition in Caco-2/15 cells.

Fatty acids	Ctl (ug/mg protein)	Fe/Asc (ug/mg protein)	AB powder+Fe/Asc(ug/mg protein)	JC-047+ Fe/Asc (ug/mg protein)
**14∶0**	6,93±0,76	4,36±0,08	5,46±0,66	7,78±0,41
**16∶0**	61,70±5,20	41,85±0,164***	55,27±7,71	70,43±6,04^###^
**18∶0**	56,14±2,04	49,57±0,41	54,7±6,36	62,88±9,35^##^
**20∶0**	1,97±0,27	1,24±0,01	2,08±0,44	2,32±0,54
**22∶0**	1,33±0,14	0,80±0,02	1,37±0,32	1,51±0,39
**24∶0**	2,50±0,30	1,32±0,01	2,55±0,78	3,08±0,79
**ALA:18∶3n-3**	0,12±0,02	0,14±0,01	0,17±0,03	0,15±0,02
**20∶3n-3**	0,07±0,02	0,12±0,03	0,13±0,04	0,16±0,09
**EPA:20∶5n-3**	3,40±0,26	1,10±0,12***	3,06±0,72^##^	3,38±1,04^###^
**22∶5n-3**	1,66±0,23	0,550±0,05	1,55±0,58	1,58±0,75
**DHA:22∶6n-3**	4,62±0,45	1,24±0,18***	4,04±1,09^##^	4,61±1,67^###^
**AL:18∶2n-6**	3,92±0,17	5,72±0,19**	4,20±0,57	4,00±0,46^#^
**18∶3n-6**	0,71±0,13	0,33±0,01	0,72±0,13	0,87±0,22
**20∶2n-6**	0,10±0,03	0,01±0,01	0,23±0,12	0,19±0,09
**20∶3n-6**	2,05±0,20	1,44±0,06	1,81±0,36	2,17±0,62
**AA:20∶4n-6**	9,55±0,81	5,76±0,66***	8,97±2,22^###^	9,42±3,13^###^
**22∶2n-6**	0,35±0,09	0,11±0,04	0,37±0,23	0,51±0,31
**22∶4n-6**	0,20±0,08	0,02±0,00	0,26±0,16	0,30±0,17
**16∶1n-7**	14,17±1,06	4,67±0,26***	12,50±1,86	15,21±0,54
**18∶1n-7**	32,09±3,47	10,83±0,31***	29,07±4,92^###^	37,10±7,47^###^
**18∶1n-9**	64,69±5,67	29,50±0,50***	60,81±10,81^###^	72,99±12,11^###^
**20∶1n-9**	4,27±0,75	1,59±0,01	4,46±1,26	5,15±1,46
**20∶3n-9**	0,63±0,03	0,33±0,05	0,56±0,09	0,58±0,09
**22∶1n-9**	10,69±3,43	3,65±0,10	4,58±0,72	4,97±1,16
**24∶1n-9**	2,59±0,43	1,03±0,04	2,86±1,35	4,16±1,81
**Total**	300.78±21.86	177.44±2.56***	274.48±43.71^###^	332.52±50.49^###^
**Total n-3**	9,87±1,32	3,15±0,484**	8,93±2,39^#^	9,88±3,51^##^
**Total n-6**	16,9±1,97	13,4±1,22	16,6±3,70	17,5±4,80
**Total n-7**	49,7±6,20	17,1±0,797***	44,5±6,90^###^	56,0±8,11^###^
**Total n-9**	82,9±13,3	36,1±0,669***	73,3±13,9^###^	87,8±15,9^###^
**Saturated FA**	137±9,58	105±0,270***	127±16,2^###^	156±18,0^###^
**Mono-unsaturated**	135±19,5	54,4±1,70***	120±21,3^###^	146±24,3^###^
**PUFA**	27,4±2,32	16,0±1,26***	26,1±6^#^	27,9±8,39^#^
**DHA/AA**	0,48±0,02	0,21±0,01**	0,44±0,02^#^	0,47±0,03^##^
**ALA/LA**	0,031±0,004	0,024±0,002**	0,039±0,003^###^	0,037±0,003^###^
**n-6/n-3**	1,73±0,04	4,29±0,19***	1,95±0,14^###^	0,17±0,04^###^

After 10 days differentiation, Caco-2/15 cells were incubated for 6 h at 37°C in the absence or presence of Fe/Asc (200 µM/2 mM) with DAPP from 250 µg/mL AB powder or JC-047 and collected for fatty acid (FA) composition. Data represent the means ± SEM of two experiments, each done in duplicate (n = 4). Student’s *t* test (two-tailed) was used to compare differences between means (X±SEM). *P<0.05, **P<0.01, ***P<0.001 vs. Ctrl; ^#^ *P*<0.05, ^##^ *P*<0.01, ^###^ *P*<0.001 vs. Fe/Asc.

AA: arachidonic acid, ALA: alpha-linolenic acid, DHA: docosahexaenoic acid, EPA: eicosapentaenoic acid, LA: linoleic acid, PUFA: polyunsaturated fatty acids.

### Mechanisms for the Action of DAPP on Oxidative Stress

As failure of antioxidant defense may explain the induction of OxS, we examined various endogenous antioxidant enzymes in Caco-2/15 cell line. Treatment with Fe/Asc alone or in combination with LPS caused a significant augmentation in the SOD activity, but preincubation of Caco-2/15 cells with the AB powder or JC-047 fraction blunted the effects of OxS and inflammation (Figure 5B). Under these conditions, GPx activity was down-regulated by Fe/Asc and LPS, and restored by treatment with the AB powder or JC-047 (Figure 5C). On the other hand, G-Red (Figure 5D) showed a trend of increase with the polyphenol treatments.

### Effects of DAPP on Inflammatory Markers

Cytokines and eicosanoids are pro-inflammatory compounds produced by the cells in response to injury. We therefore assessed the production of TNF-α and IL-6, two powerful inflammatory biomarkers, in Caco-2/15 cells incubated with Fe/Asc, LPS or their combination for 6 h. Analysis by Western Blot disclosed an elevation of protein mass of TNF-α (1.5 to 2.0-fold) and IL-6 (1.5 to 1.8-fold) in the presence of Fe/Asc and LPS, respectively, compared to control cells (Figure 6). Pre-treatment with the AB powder or JC-047 fraction abolished the increase in TNF-α and IL-6 protein expression in Caco-2/15 cell line.

**Figure 6:** Effects of DAPP on oxidative stress or LPS-induced inflammation on inflammatory markers in Caco-2/15 cells. Crude AB powder (250 µg/mL) and purified JC-047 fraction (250 µg/mL) were added to the apical compartment of differentiated Caco-2/15 cells for 24 h before incubation with Fe/Asc (200 µM/2 mM) and LPS (200 µg/mL) for 6 h at 37°C as described in Materials and Methods. Protein expression of the inflammatory markers TNF-α (A to C) and IL-6 (D to F) was determined by Western blot, respectively. Results represent the means ± SEM of n = 3 independent experiments. *P<0.05, **P<0.01, ***P<0.001 vs. Ctrl; ^###^ *P*<0.001 vs. Fe/Asc;^ †^ *P*<0.05, ^†††^ *P*<0.001 vs. LPS; ^$$$^ *P*<0.001 vs. Fe/Asc+LPS.

We next turned to the formation of inflammatory eicosanoids such as PGE2 that is synthesized from arachidonic acid by COX-2. Our experiments showed that Fe/Asc and LPS elicited exaggerated synthesis of PGE2 whereas preincubation with the AB powder displayed high ability to prevent PGE2 accumulation in response to LPS but not Fe/Asc (Figure 6).

### Mechanisms for the Action of DAPP on Inflammation

Since the COX-2 enzyme may be behind the elevation of Fe/Asc- and LPS-induced PGE2, we determined its protein expression. Both stimuli raised its protein mass as evidenced by Western blot (Figure 7). Pre-incubation of Caco-2/15 cells with the AB powder or JC-047 fraction averted the positive action of the oxidative and inflammatory stimuli on COX-2 protein expression. Importantly, the polyphenol antioxidants were as effective as indomethacin heptyl ester, a selective COX-2 inhibitor [45] in preventing the elevation of PGE2. In addition, their combination provided a more substantial synergetic effect, which is indicative of different mechanisms of action for LPS-induced inflammation (Figure 8).

**Figure 7:** Effects of DAPP on oxidative stress and LPS-induced inflammation on prostaglandin E2 in Caco-2/15 cells. Crude AB powder (250 µg/mL) and purified JC-047 fraction (250 µg/mL) were added to the apical compartment of differentiated Caco-2/15 cells for 24 h before incubation with Fe/Asc (200 µM/2 mM) and LPS (200 µg/mL) (A), as well as indomethacin heptyl ester (0.4 µM) (B), as a selective cyclooxygenase (COX)-2 inhibitor, for 6 h at 37°C as described in Materials and Methods. PGE2 was determined by enzymatic immunoassay. Results represent the means ± SEM of N = 3 independent experiments. ***P<0.001 vs. Ctrl; ^†††^ *P*<0.001 vs. LPS; ^$$$^ *P*<0.001 vs Fe/Asc+LPS.

**Figure 8:** Effects of DAPP on oxidative stress or LPS-induced inflammation on cyclooxygenase 2 modulation in Caco-2/15 cells. Crude AB powder (250 µg/mL) and purified JC-047 fraction (250 µg/mL) were added to the apical compartment of differentiated Caco-2/15 cells for 24 h before incubation with Fe/Asc (200 µM/2 mM) and LPS (200 µg/mL) (A to C), as well as indomethacin heptyl ester (0.4 µM) (D), as a selective cyclooxygenase (COX)-2 inhibitor, for 6 h at 37°C as described in Materials and Methods. Protein expression of COX-2 was determined by Western blotting. Results represent the means ± SEM of n = 3 independent experiments. **P<0.01, ***P<0.001 vs. Ctrl; ^###^ *P*<0.001 vs. Fe/Asc; ^††^ *P*<0.01, ^†††^ *P*<0.001 vs. LPS; ^$$$^ *P*<0.001 vs Fe/Asc+LPS.

### Mechanisms for the Action of DAPP on Transcription Factors

NF-κB signaling pathway plays a crucial role in the initiation and amplification of inflammation via the modulation of multiple inflammatory mediators. Figure 9 shows that Caco-2/15 cells exposed to Fe/Asc or LPS displayed a high NF-κB signal in the nucleus along with a low level of IκB protein expression in the cytoplasm, which suggests that the inhibitory protein is degraded by the proteasome, leaving NF-κB free to enter the nucleus and activate the transcription of its target genes. As a consequence, the NF-κB/IκB ratio was increased under the presence of Fe/Asc (Figure 9A) and LPS (Figure 9B and 7C). Importantly, the AB powder or JC-047 fraction displayed their great potential to neutralize IκB degradation and NF-κB mobilization to the nucleus compared to CAPE, the NF-κB inhibitor, with LPS at 6 h (Figure 9B) and LPS at 24 h (Figure 9C) to mimic an acute and a long inflammation, respectively. The combined administration of CAPE and AB powder or JC-047 fraction did not produce significant changes, thereby indicating the same mechanisms of action.

**Figure 9:** Effects of DAPP on oxidative stress or LPS-induced inflammation on NF-κB in Caco-2/15 cells. Crude AB powder (250 µg/mL) and purified JC-047 fraction (250 µg/mL) in the presence or absence of 50 µM caffeic acid (CAPE, a specific NF-κB inhibitor) were added to the apical compartment of differentiated Caco-2/15 cells for 24 h before incubation with Fe/Asc (200 µM/2 mM) (A) and LPS (200 µg/mL) (B) for 6 h at 37°C, and LPS (200 µg/mL) (C) for 24 h at 37°C to mimic a chronic inflammation as described in Materials and Methods. Results represent the means ± SEM of n = 3 independent experiments. **P<0.01, ***P<0.001 vs. Ctrl;^ #^ *P*<0.05, ^##^ *P*<0.01, ^###^ *P*<0.001 vs. Fe/Asc; ^†††^ *P*<0.001 vs. LPS.

To decipher the mechanisms of action of the AB powder or JC-047 fraction, we examined the transcription factors that are involved in the regulation of antioxidant genes expression. The protein mass of Nrf2 in homogenates (Figure 10A) and nuclei (Figure 10B) was down-regulated by Fe/Asc- or LPS-induced OxS and inflammation, respectively. However, treatment with the AB powder or JC-047 fraction restored Nrf2 protein expression to the basal level. We also assessed the protein expression of PGC-1α a powerful transcriptional co-activator that up-regulates Nrf2. PGC-1α protein mass was down-regulated in response to OxS and inflammation in homogenates (Figure 10C) and nuclei (Figure 10D) in Caco-2/15 cells. However, the effect was reestablished when Caco-2/15 cells were pre-incubated with the AB powder or JC-047 fraction.

**Figure 10:** Effects of DAPP oxidative stress or LPS-induced inflammation on transcription factors in Caco-2/15 cells. AB powder (250 µg/mL) and purified JC-047 fraction (250 µg/mL) were added to the apical compartment of differentiated Caco-2/15 cells for 24 h before incubation with Fe/Asc (200 µM/2 mM) and LPS (200 µg/mL) for 6 h at 37°C as described in Materials and Methods. Protein expression of the transcription factors Nrf2 in homogenates (A) and in nucleus (B), as well as PGC-1α in homogenates (C) and in nucleus (D) was determined by Western blot. Results represent the means ± SEM of n = 3 independent experiments. *P<0.05, **P<0.01, ***P<0.001 vs. Ctrl; ^#^ *P*<0.05, ^##^ *P*<0.01, ^###^ *P*<0.001 vs. Fe/Asc; ^$^ *P*<0.05, ^$$^ *P*<0.01, ^$$$^ *P*<0.001 vs. Fe/Asc+LPS.

## Discussion

Growing evidence suggests important roles of dietary factors in preserving health and even reversing the progression of chronic diseases, with anti-inflammatory effects as important underlying mechanisms. In the present study, we first characterize the polyphenol compounds of DAPP by HPLC-ESI-MS TOF and then tested their impact on cell integrity and viability. After we excluded any possible toxicity of this natural DAPP (crude extract) and its purified fraction, which has frequently been detected in various chemical drugs, we could subsequently document their remarkable capacity in scavenging ROS and neutralizing inflammation in intestinal absorptive cells. By dissecting the mechanisms of action, our *in vitro* experiments highlighted the ability of apple peel polyphenols to increase the antioxidant/anti-inflammatory defense by (i) preventing LPS-induced inflammation via limitation of the pro-inflammatory expression and activity of COX-2; (ii) ruling out LPS-mediated cytokine production through downregulation of NF-κB, an essential transcription factor for numerous cytokines and (iii) up-regulating the expression of transcription factors (Nrf2 and PGC-1α), key redox-sensitive transcription factors and crucial elements for mitochondrial biogenesis.

The results of our comprehensive study provide fundamental information on the apple peel polyphenols. The high-resolution HPLC-ESI-MS TOF delivers the composition of the different biomolecules in DAPP (AB powder or JC-047 fraction). In the former, flavonols (composed of aglycone and glycosylated quercetin and dihydrochalcone) are the major subclasses of flavonoids present, while in the purified fraction, we mostly found the flavan-3-ols and their oligomers. Noteworthy, quercetin represents the preponderant flavonol in DAPP and, according to previous studies; it has exhibited anti-inflammatory and antioxidant activities, prevented platelet aggregation and promoted relaxation of cardiovascular smooth muscle [46]. As a matter of fact, flavan-3-ols are a family of bioactive compounds and potent antioxidants as has been described in *in vitro* and *in vivo* studies. Importantly, in the current work, we have evaluated the antioxidant and anti-inflammation power of both the crude extract (AB powder) and purified polyphenol fraction (JC-047) derived from DAPP since there was a need to prove that the beneficial effects are derived from the polyphenos contained in apple peels.

In the present work, we used the Caco-2/15 cell line that undergoes a process of spontaneous differentiation leading to the formation of a monolayer of cells expressing several morphological and functional characteristics of the mature enterocyte. This remarkable intestinal model is regarded as the most appropriate for the investigation of gut absorption and interactions, nutrition, toxicology food microbiology, bioavailability tests, and screening of drug permeability in discovery programs. Multiple studies from our laboratory have shown that Caco-2/15 cell monolayers are fully appropriate for the study of OxS and inflammation [38], [39], [41], [47].

To produce OxS, we employed the Fe/Asc complex, a widely used oxygen-radical generating system [34], [36], [39], [41], [42] since our laboratory reported the ability of iron to initiate strong lipid peroxidation, whereas ascorbic acid can amplify iron-oxidative potential by promoting metal ion-induced lipid peroxidation [34]. The data of the present study clearly indicate that the Fe/Asc system functioned as a producer of lipid peroxidation given the production of MDA and the degradation of PUFAs and the production of pro-inflammatory eicosanoids. Additionally, with the Fe/Asc complex, the antioxidant/oxidative balance deteriorated the endogenous antioxidant enzymes. In this context, co-supplementation of iron and vitamin C worsens OxS in the gastrointestinal tract, thereby leading to ulceration in healthy individuals, and exacerbates chronic gastrointestinal inflammatory diseases, which may result in the development of cancers [48]. Importantly, supplementation of DAPP by crude extract or its purified fraction significantly prevented lipid peroxidation and restored the depletion of some n-3 PUFA, likely by strengthening the endogenous antioxidant defense as illustrated, in our results, through SOD down-regulation and GPx up-regulation activities.

For the induction of inflammation, we used LPS that has been extensively studied for the past two decades. This is a ubiquitous endotoxin mediator of gram-negative bacteria, which facilitates microbial translocation by a mechanism implicating physical perturbation of the gut mucosal barrier [1], [49]. LPS is also a potent inducer of the host’s immune response via its capacity to stimulate the pro-inflammatory cytokine cascade. In our studies, LPS led to amplification of the inflammatory response in Caco-2/15 cells given the enhanced production of PGE2 and the raised protein expression of TNF-α and IL-6, probably due to elevated COX-2 and NF-κB, respectively. DAPP was effective in preventing the elevation of PGE2, TNF-α and IL-6 via the down-regulation of COX-2 and NF-κB, as evidenced by the co-administration of their specific inhibitors indomethacin heptyl ester and CAPE, respectively. The combination of CAPE and DAPP (either as crude extract or its purified JC-047 fraction) did not further anti-inflammatory benefits, which suggests a common mechanism of action. On the other hand, compounding indomethacin heptyl ester and DAPP resulted in amplified anti-inflammatory effects, which argues in favor of synergetic mechanisms.

Since the Keap1-Nrf2-antioxidant response element (ARE) is an integrated redox sensitive signaling system that regulates from 1% to 10% of our genes [50], [51], we assessed the protein expression of Nrf2 and could document its significant increase. It is therefore possible that, upon exposure to AB powder or JC-047 fraction, Nrf2 was able to escape Keap1-mediated ubiquitin-dependent proteasomal degradation, translocate to the nucleus, and activate ARE-dependent gene expression of a series of antioxidative and cytoprotective proteins that include SOD and GPx. Our study went even further since it revealed the positive modulation of PGC-1α by DAPP. PGC-1α controls many aspects of oxidative metabolism, including mitochondrial biogenesis and respiration through the coactivation of many nuclear receptors [52], [53]. As an example, Nrf2 is a key target of the PGC-1α in mitochondrial biogenesis and important protective molecules against ROS generation and damage. It is therefore possible that PGC-1α activates NRF2 to induce the SOD and GPx that were altered by Fe/Asc-mediated lipid peroxidation. However, additional efforts are needed to understand the role of DAPP in PGC-1α and Nrf2 cross-talk.

Noteworthy, in some experiments, Caco-2/15 cells were serum-starved for 24 h prior to the addition OxS or inflammation. The serum-depleted media were used to minimize the formation of adducts between DAPP and serum proteins, and to exclude the interferences originating from available factors present in fetal bovine serum, as described in previous studies with other types of antioxidants [54]. The pre-incubation time of 24 h with DAPP was used to maximally strengthen the antioxidant and anti-inflammatory defense before the addition of the iron-ascorbate oxygen radical-generating system or LPS that triggers inflammation. By allocating this period of time, we allow Caco-2/15 cells to deploy various powerful protection mechanisms via transcription factors and signaling pathways. The transport and processing of DAPP have been elaborated in the Discussion section.

Following their consumption, polyphenols are extensively metabolized by hydrolyzing and conjugating enzymes [55], [56]. They are first conjugated in the small intestine to form O-glucuronides, sulphate esters and O-methyl ether [57] before reaching the liver for further metabolism [58]. The formation of anionic derivatives by conjugation with glucuronides and sulphate groups facilitates their urinary and biliary excretion and explains their rapid elimination. Non-absorbed polyphenols and the fraction re-excreted by the bile are extensively metabolized and transformed by the microbiota before absorption [59], [60]. The transformation by commensal bacteria via esterase, glucosidase, demethylation, dehydroxylation, and decarboxylation is often essential for absorption and modulates the biological activity of these polyphenols [60]. In our intestinal model, no flora is present, which suggests an absorption via paracellular route of transport as suggested previously [61]. However, additional studies are still needed to highlight the contribution of trans-membrane vs. intercellular absorption as well as the influence of polyphenols of enterocyte metabolism just by adherence to the brush border membrane.

Previous studies investigated the preventive effectiveness of polyphenolic content of flesh apple in cultured gastric mucous cells under conditions independent of acid secretion or systemic factors [62]. They identified the composition of phenolic compounds (chlorogenic acid, caffeic acid, catechin, epicatechin, rutin and phloridizin) in apple flesh extracts, which prevented OxS-induced injury to gastric epithelial cells by permeating cell membranes, increasing intracellular antioxidant activity, and inhibiting ROS-dependent lipid peroxidation. In further studies, the same apple flesh extracts demonstrated prevention of aspirin-induced damage to the rat gastric mucosa [63] and an anti-inflammatory effect on colonic injury in rats with trinitrobenzensulphonic acid-induced colitis [64]. Even though these reports with apple flesh extracts, and ours with DAPP show anti-inflammatory and antioxidant effects, it is not possible to compare their effectiveness given the differences in the apple species, extraction methodology, experimental models and techniques.

In conclusion, a plethora of studies demonstrates significant health benefits of nutrient rich fruits. If various studies have shown this relationship by indirect evidences, the present work demonstrated the presence of a nonpolar bioactivity in extracts of DAPP and their direct beneficial actions, which negated operational OxS and inflammation, both elicited by state-of-the-art techniques. Our results suggest that DAPP may represent a new strategy for the prevention of OxS and inflammation associated with IBD. Further studies are needed to investigate this hypothesis.
